# Histology and molecular pathology of iliotibial tract contracture in patients with gluteal muscle contracture

**DOI:** 10.1042/BSR20181351

**Published:** 2019-09-20

**Authors:** Bang-tuo Yuan, Feng Qu, Shao-xia Wang, Wei Qi, Xue-zhen Shen, Chun-bao Li, Yu-jie Liu

**Affiliations:** 1 Department of Orthopedics, Tianjin Hospital, Tianjin 300211, China; 2 Department of Orthopedics, Beijing Tongren Hospital, Capital Medical University, Beijing 100730, China; 3 Institute of Radiation Medicine, Academy of Military Medical Sciences, Beijing 100850, China; 4 Department of Orthopedics, the First Medical Center, Chinese PLA General Hospital, Beijing 100853, China

**Keywords:** contracture, gluteal muscles, iliotibial tract, molecular pathology, tissue repair

## Abstract

The present study aimed to examine the pathologic changes of the iliotibial tract and discusses its relationship with gluteal muscle contracture. Samples of contractual iliotibial tracts were collected from six patients with contractures of the gluteal muscles and iliotibial tracts during their surgical treatment. Samples of normal iliotibial tracts were collected from six patients receiving surgeries for avascular necrosis of the femoral head who had no contractures of the gluteal muscles and iliotibial tracts. The tissue samples were stained using Hematoxylin and Eosin (H&E), Masson’s trichrome, and Sirius Red. The mRNA and protein levels of various tissue repair genes were determined using quantitative real-time PCR and Western blotting. Both the normal and contractual iliotibial tracts consisted of type I and III collagens. The contractual iliotibial tracts had a significantly higher proportion of type III collagen in comparison with the normal iliotibial tracts. The mRNA expression levels and protein levels of tissue repair genes TGFβ 1, bFGF, and matrix metalloproteinase-1 (MMP-1) in the contractual iliotibial tracts were up-regulated in comparison with that in the normal iliotibial tracts. However, the mRNA expression levels and protein levels of tissue inhibitors of metalloproteinase-1 (TIMP) in the contractual iliotibial tracts were down-regulated in comparison with that in the normal iliotibial tracts. The contractures of both the gluteal muscles and the iliotibial tracts share similar histology and molecular pathology. Our results indicate that iliotibial tract contracture is secondary to the gluteal muscle contracture and is a constant tissue repair process.

## Introduction

Gluteal muscle contracture is a clinical syndrome caused by fibrosis and necrosis of the gluteal muscles and fasciae. Its symptoms include restricted hip movement, awkward gait, anterior knee pain, and limb deformity [1–3], which are caused by hip adduction and internal thigh rotation [4]. Repeated intramuscular injections at a younger age are thought to be the most important etiology of gluteal muscle contracture [5–11], although other mechanisms, such as immunology and genetics, may also play roles in the development of this disease.

Earlier 2% benzyl alcohol was widely used as solvent for penicillin as a measure to ease the injection pain in children in China. Benzyl alcohol is a weak local anesthetic and preservative. However, the combination of benzyl alcohol and penicillin causes strong stimulation in the muscle, which can cause in hemolysis and immune reactions. This leads to local ischemia and hypoxia, and finally the initiation of tissue repair. Another theory is that rapid injection of fluid into the muscles causes local compression and ischemia, leading to tissue repair. During tissue repair, the fibroblasts significantly proliferates and migrates (with possible differentiation), and secrets large amounts of type I and III collagens and multiple proteins. This process is also accompanied with the activation of many cytokines and signaling pathways. For example, there is evidence that the TGF-β/Smad signaling pathway plays a role in the development of gluteal muscle contraction [12]. In addition, FGFs are key players in skeletal muscle regeneration, with bFGF playing an essential role after injury [13]. It is also recognized that the overproduction and deposition of collagens and tissue remodeling is regulated by matrix metalloproteinases (MMPs) and their physiological inhibitors, tissue inhibitor of metalloproteinases (TIMPs) [14]. In particular, MMP-1 cleaves the triple helix of interstitial collagen types I, II, and III, and TIMP-1 is the natural inhibitor of both collagenase I and gelatinase [15]. MMP-1-treated muscle cells show an increased migration and myogenic differentiation capacity [16], and in skeletal muscles, TIMP-1 is up-regulated and is involved in cell fusion [17]. All these changes result in apoptosis and pathological tissue remodeling, leading to excessive collagens in the muscular lesion and finally the muscular contracture.

Many patients with gluteal muscle contracture also had contractual iliotibial tract [18]. The presence of contractures in both the gluteal muscles and the iliotibial tracts suggest that they may share the same pathologic mechanisms. The present study aimed to examine the pathologic changes and molecular mechanisms involved in the iliotibial tract contracture in patients with gluteal muscle contracture.

## Materials and methods

### Patients

The samples (1.5 × 1.0 × 0.5 cm) of contractual iliotibial tracts were collected intraoperatively from six patients receiving surgical release of contractures of the gluteal muscles and the iliotibial tracts. The samples (1.5 × 1.0 × 0.5 cm) of normal iliotibial tracts were collected intraoperatively from six patients receiving surgeries for avascular necrosis of the femoral head who had no contractures of the gluteal muscles and iliotibial tracts. The tissue specimens were selected from the iliac crest of the femoral greater trochanter. The iliotibial bundle at the proximal end of the margins were selected as the experimental specimen. The tissue around the surgical microscope is rough and generally trimmed—the sizes were approximately 1.5 cm long, 1 cm wide, and 0.5 cm thick. Patient demographics are elaborated in Table 1. Our study was approved by our institutional ethics committee. Informed consent was obtained from each participant.

**Table 1:** Demographics of patients included in the current study

Normal iliotibial tracts (*n*=6)	
Age	65.33 ± 5.32 years
Gender	
Male	50%
Female	50%
History of intramuscular injection	No
Contractual iliotibial tracts (*n*=6)	
Age	27.67 ± 2.42 years
Gender	
Male	50%
Female	50%
History of intramuscular injection	
Kind of injection	Penicillin in 2% benzyl alcohol as solvent
Initial age at administration	14.17 ± 2.32 months
Number of injections	15 ± 3.4

### Staining

The tissue blocks were fixed in 10% formalin at room temperature for 72 h. After dehydration and clearing, the tissue blocks were paraffin-embedded and cut into 3-μm sections. The sections were stained using Hematoxylin and Eosin (H&E) to examine the general histology of the iliotibial tracts. Masson’s trichrome staining and Sirius Red staining were used to examine the collagen fibers. The Sirius Red-stained sections were observed using a polarizing microscope. Section pictures were taken using a digital camera and analyzed.

### Staining and image analysis

The tissue sections were stained with Masson’s trichrome or Sirius Red and were imaged at 200× magnification using bright light microscopy. For the Sirius Red staining, the sections were also imaged using polarized light microscopy to show the type I collagen in red and the type III collagen in green. For each patient, five sections were selected and ten vision fields were imaged for each section. Using the stained images, the collagen density was measured using the CMIAS-II image analyzing system.

### Quantitative real-time PCR

The samples of iliotibial tracts were collected intraoperatively and immediately put into liquid nitrogen. The RNA was extracted using the TRIzol method and reversely transcribed into cDNA. The same amount of starting cDNA was used for all of the reactions. The real-time PCR consisted of 1 cycle of 2 min at 50°C, 1 cycle of 1 min at 90°C, 40 cycles of 15 s at 95°C and 1 min at 60°C, 15 s at 95°C, 30 s at 60°C, and 1 cycle of 30 s at 95°C. The sequences of primers are listed in Table 2. *HPRT1* was used as the reference gene. The changes in gene expression was calculated as 2^−ΔΔ*C*^_t_. Δ*C*_t_ = *C*_t_ (target gene) – *C*_t_ (reference gene).

**Table 2:** Primers used in the current study

	Forward (5′–3′)	Reverse (5′–3′)
*TGFβ1*	ACCTGAACCCGTGTTGCTCT	CTAAGGCGAAAGCCCTCAAT
*bFGF*	GGCTTCTTCCTGCGCATCCAT	GGTAACGGTTAGCACACACTCCTTT
*MMP1*	CTGGCCACAACTGCCAAATG	CTGTCCCTGAACAGCCCAGTACTTA
*TIMP1*	TGCACCTGTGTCCCACCCCACCC	TGGGACCGCAGGGACTGCCAGGT
*HPRT1*	CATTATGCTGAGGATTTGGAAAGG	CTTGAGCACACAGAGGGCTACA

Abbreviations: HPRT1, hypoxanthine phosphoribosyltransferase 1; TGF-β1, transforming growth factor β 1.

### Western blotting

The total protein was extracted from the frozen tissue blocks. Forty micrograms of the sample protein from each tissue was electrophoresed and transferred on to a PVDF membrane. The PVDF membrane was incubated with primary antibodies at 4°C overnight (Table 3). Goat-anti rabbit secondary antibody (1:2000, CWBio, Beijing, China) was added on to the membrane for 1 h. The blot was Coomassie stained and used for densitometric analysis using the Labwork software.

**Table 3:** Primary antibodies used in the current study

Antibody	Species	Dilution	Producer
TGF-β1	Rabbit	1:1000	Cell Signaling Technology, U.S.A.
bFGF	Rabbit	1:1000	Abcam, U.K.
MMP-1	Rabbit	1:5000	Abcam, U.K.
TIMP-1	Rabbit	1:1000	Cell Signaling Technology, U.S.A.

Abbreviations: TGF-β1, transforming growth factor β 1.

### Statistical analysis

All data were expressed as mean ± standard deviation and compared using Student’s *t* test or rank-sum test. All statistical analyses were performed using the SPSS 22.0 software. A *P*-value less than 0.05 was considered statistically significant.

## Results

### H&E staining

H&E staining showed that the connective tissue in normal iliotibial tracts was regularly and consistently arranged (Figure 1A). However, connective tissue from the contractual iliotibial tracts had a disrupted structure and arrangement (Figure 1B).

**Figure 1:** H&E staining H&E staining of the normal iliotibial tracts (**A**) and the contractual iliotibial tracts (**B**). Scale bar, 100 μm.

### Collagen staining

The Masson’s trichrome staining showed that the normal iliotibial tracts consisted of bundles of collagen fibers, which were in a tight arrangement (Figure 2A). In the contractual iliotibial tracts, the collagen fibers were in a wave-like format with wider gaps (Figure 2B). Quantification of the staining by the CMIAS-II image analyzing system revealed that the collagen density in the contractual iliotibial tracts was significantly lower than in the normal iliotibial tracts (0.8604 ± 0.0198 vs 0.9051 ± 0.0110, *P*=0.002).

**Figure 2:** Masson’s trichrome staining Masson’s trichrome staining of the normal iliotibial tracts (**A**) and the contractual iliotibial tracts (**B**). Scale bar, 100 μm.

The Sirius Red staining showed that the normal iliotibial tracts were positive for collagen fibers by bright light microscopy, and the polarized light microscopy showed that it primarily consisted of type I collagen and a minimal amount of type III collagen (Figure 3A,B). In contrast, in the contractual iliotibial tracts, by bright light microscopy, the fiber density decreased and by the polarized light microscopy showed that the proportion of type III collagen was significantly increased (Figure 3C,D). The quantification of the staining by the CMIAS-II image analyzing system revealed that the collagen density in the contractual iliotibial tracts was significantly lower than in the normal iliotibial tracts (0.8241 ± 0.0379 vs 0.9220 ± 0.0152, *P*=0.001).

**Figure 3:** Sirius Red staining The normal iliotibial tracts (**A,B**) primarily consisted of type I collagen (red) and a small amount of type III collagen (green). In the contractual iliotibial tracts (**C,D**), the proportion of type III collagen (green) was significantly increased. Scale bar, 50 μm.

### mRNA expression levels of tissue repair genes

The mRNA expression levels of *TGFB1, bFGF*, and *MMP1* in the contractual iliotibial tracts were significantly up-regulated in comparison with that in the normal iliotibial tracts. However, the mRNA expression levels of *TIMP1* in the contractual iliotibial tracts were significantly down-regulated in comparison with that in the normal iliotibial tracts (Figure 4).

**Figure 4:** The differential expression of tissue repair genes in the normal and contractual iliotibial tracts Data were normalized to *HPRT1* and expressed as mean ± standard deviation of three independent experiments. Abbreviations: bFGF, basic fibroblast growth factor; HPRT1, hypoxanthine phosphoribosyltransferase 1; MMP1, matrix metalloproteinase-1; TIMP1, tissue inhibitor of metalloproteinase-1; TGF-β1, transforming growth factor β 1. *P<0.05.

### Protein levels of tissue repair genes

The protein levels of TGFβ-1, bFGF, and MMP-1 in the contractual iliotibial tracts were significantly higher than that in the normal iliotibial tracts (Figure 5A,B, *P*<0.05). However, the protein levels of TIMP-1 in the contractual iliotibial tracts were significantly lower than that in the normal iliotibial tracts (Figure 5A,B, *P*<0.05).

**Figure 5:** Relative protein expression of indicated candidates in normal (*N*) and contractual (*C*) iliotibial tract, respectively (**A**) Shown are representative blot. The blot was stained with Coomassie stain to ensure equal protein loading. (**B**) Densitometric analysis of relative protein expression of indicated candidates from three independent experiments. Data were normalized to total protein expression and expressed as mean ± standard deviation. Abbreviations: bFGF, basic fibroblast growth factor; MMP-1, matrix metalloproteinase-1; TGF-β1, transforming growth factor β 1; TIMP-1, tissue inhibitor of metalloproteinase-1. *P<0.05.

## Discussion

The gluteus maximus is a coarsely fasciculated muscle that lies in the superficial portion of the buttock. It is quadrilateral, and its fasciculi are oriented downward and outward. The gluteus maximus emerges from the posterior gluteal line of the ilium and the area of the bone above and behind it, the posterior surface of the sacrum and coccyx, the sacrotuberal ligament and the gluteal aponeurosis overlying the gluteus medius muscle. The superficial fibers and the larger upper portion of the muscle of the lower portion are embedded into the iliotibial tract of the fascia lata. The deeper fibers of the muscle in the lower portion reach the gluteal tuberosity of the femur and the lateral intermuscular septum [19]. Fibrous muscular contracture, including gluteal contracture, is diagnosed clinically by the characteristic physical deformities and limited motions of the adjacent joint or limb [20]. Iliotibial tract contracture is a frequent complication in patients with contractual gluteal muscles caused by frequent intramuscular injections at a younger age. Our study found that the contractual iliotibial tracts in these patients had similar pathological changes with that of the contractual gluteal muscles.

To examine the histology of the contractual iliotibial tracts, we used H&E staining, Masson’s trichrome staining, and Sirius Red staining. Masson’s trichrome staining can reveal the general distribution and changes in collagens, giving an overall view of the fibrosis in the lesions as wells as its boundary in the muscles. However, Masson’s trichrome staining is unable to distinguish the different types of collagen, which is the reason for the use of Sirius Red staining. By using Sirius Red staining with polarized light microscopy, the mature and thick type I collagen are in bright yellow or red colors, while the fresh and thin type III collagen are in green color. Our study found that both the normal and contractual iliotibial tracts are composed of fibrous connective tissue. H&E and Masson’s trichrome staining showed that the contractual iliotibial tracts had disarranged and tortuous structures. Sirius Red staining showed that although normal and contractual iliotibial tracts had type I and III collagens, the latter had a significantly higher proportion of type III collagen in comparison with the normal ones.

Type III collagen is fresh and thin, and usually is secreted in large amount in the early stage of tissue repair [21]. The mature and thick type I collagen replaces type III collagen in the late stage of tissue repair, thus increasing the hardness of the scar tissue. The large amount of type III collagen in the contractual iliotibial tracts in our patients suggested that there is continuous tissue repair in the lesions [22]. Since the intramuscular injections that cause the gluteal muscle contractures occurred many years ago, our results indicated that the iliotibial tract contracture is secondary to the gluteal muscle contracture. Gluteal muscle contracture may increase the tension of the iliotibial tract, resulting in persistent injury and repair. This finally leads to the pathological proliferation and thickening of the iliotibial tracts.

To understand the molecular pathology in the contractual iliotibial tracts, we examined the mRNA expression levels and the protein levels of six tissue repair genes. Our study found that the mRNA expression levels and protein levels of TGF-β1, bFGF, and MMP-1 in the contractual iliotibial tracts were up-regulated in comparison with that in the normal iliotibial tracts. However, the mRNA expression levels and protein levels of TIMP-1 in the contractual iliotibial tracts were down-regulated in comparison with that in the normal iliotibial tracts.

TGF-β1 up-regulates the expression of collagen genes in the fibroblasts, which explains the large amounts of collagens in the contractual iliotibial tracts. In addition, TGF-1β1 induces differentiation from the fibroblasts to the myofibroblasts [23]. The myofibroblasts can cause wound contraction during the process of tissue repair [24]. The persistence of myofibroblasts is a mark of fibrosis and scar tissue. This may also cause the corresponding clinical symptoms in our patients with iliotibial tract contractures.

bFGF is a member of the fibroblast growth factor family. In addition, to promote the proliferation of fibroblasts, bFGF can also induce the migration of endothelial cells, Keratinocytes, vascular smooth muscle cells, and fibroblasts [25–27]. Fibroblasts are the primary target cells of bFGF during tissue repair. bFGF influences the proliferation and migration of fibroblasts, increases the expression of fibronectin and MMP-1, and disturbs the distribution of collagens. Therefore, bFGF plays important roles in tissue repair. Our study found that bFGF was up-regulated at both mRNA and protein levels in the contractual iliotibial tracts in comparison with that of normal iliotibial tracts. In the contractual iliotibial tracts, the normal collagens are significantly degenerated and the tissue is in constant damage and repair. The up-regulation of bFGF may accelerate the process of tissue repair in the contractual iliotibial tracts.

MMP-1 is a well-known MMP. TIMP-1 is an endogenous inhibitor of MMPs, and is secreted by activated fibroblasts and endothelial cells. The dynamic balance of MMP-1/TIMP-1 is critical in maintaining extracellular matrix levels. Our study found that MMP-1 was up-regulated and TIMP-1 was down-regulated at both mRNA and protein levels in the contractual iliotibial tracts in comparison with that in the normal iliotibial tracts. These findings were consistent with regenerated and/or repaired tissues.

## Conclusions

Patients with gluteal muscle contractures often also have contractual iliotibial tracts. The contractures of both the gluteal muscles and the iliotibial tracts share similar histology and molecular pathology. There is a high proportion of type III collagen in the contractual iliotibial tracts, suggesting that iliotibial tract contracture is secondary to the gluteal muscle contracture and is a constant tissue repair process. Various tissue repair genes are involved in the pathology of iliotibial tract contractures.

## Abbreviations

bFGF: basic fibroblast growth factor
H&E: Hematoxylin and Eosin
HPRT1: hypoxanthine phosphoribosyltransferase 1
MMP: matrix metalloproteinase
TGF-β: transforming growth factor β
TIMP: tissue inhibitor of metalloproteinase
